# Continuous Incisional Lidocaine in Pediatric Patients following Open Heart Surgery

**DOI:** 10.1155/2022/1403539

**Published:** 2022-01-04

**Authors:** Sarah Nicole Fernández, Blanca Toledo, Jesús Cebrián, Ramón Pérez-Caballero, Jesús López-Herce, Santiago Mencía

**Affiliations:** ^1^Department of Paediatric Intensive Care, Hospital General Universitario Gregorio Marañón, Madrid, Spain; ^2^Complutense University of Madrid, Spain. School of Medicine. Department of Pediatrics, Spain; ^3^Health Research Institute of the Gregorio Marañón Hospital, Madrid, Spain; ^4^Department of Anesthesiology, Hospital General Universitario Gregorio Marañón, Madrid, Spain; ^5^Department of Pediatric Heart Surgery, Hospital General Universitario Gregorio Marañón, Madrid, Spain

## Abstract

Continuous incisional lidocaine infusion has been proposed as an adjunctive therapy in the management of postoperative pain in adult patients. The aim of this study was to determine the efficacy and safety of a continuous subcutaneous lidocaine infusion in pediatric patients following open heart surgery. All patients receiving a subcutaneous lidocaine infusion in median sternotomy incisions after open heart surgery during 2 consecutive years were included in the study. A historical cohort of patients was used as a control group. Demographic variables (age, size, and surgical procedure), variables related to sedation and analgesia (COMFORT and analgesia scales, drug doses, and duration), and complications were registered. 106 patients in the lidocaine infusion group and 79 patients in the control group were included. Incisional analgesia was effective for the treatment of pain as it reduced the dose and duration of intravenous fentanyl (odds ratio (OR) 6.26, confidence interval (CI) 95%: 2.48-15.97, *p* = 0.001; OR 4.30, CI 95%: 2.09-8.84, *p* = 0.001, respectively). The reduction in fentanyl use was more important in children over two years of age. Adverse effects were seen in three children (2.8%): they all had decreased level of consciousness, and one of them presented seizures as well. Two of these three patients had lidocaine levels over 2 mcg/ml. A continuous lidocaine incisional infusion is effective for the treatment of pain after open heart surgery. This procedure reduced intravenous analgesic drug requirements in pediatric patients undergoing a median sternotomy incision. Although the incidence of secondary effects is low, monitoring of neurologic status and lidocaine blood levels are recommended in all patients.

## 1. Introduction

Appropriate analgesia after a surgical intervention is essential, especially after sternotomy in pediatric patients [1–5].

Pain management in the postoperative period includes intravenous analgesic drugs such as opioids, nonsteroidal anti-inflammatory drugs, metamizole, and paracetamol [3, 4]. Over the few last years, however, some authors have recommended a multimodal approach combining intravenous drugs with regional techniques such as epidural analgesia, nerve block, or continuous infusion of local anaesthesia into the surgical wound [2, 5–10] in order to improve analgesic efficacy and to decrease adverse effects [1–3, 11].

Incisional analgesic infusion consists of a continuous administration of a local anaesthetic in the subcutaneous tissue of the surgical wound through a catheter placed during the surgical procedure [12–16]. Several studies performed in adults show the efficacy of incisional analgesia to decrease postoperative pain in different kinds of surgeries, including open heart surgery [1, 12–14, 16]. However, there is limited evidence about its use in pediatric patients [15–17].

The aim of our study is to determine the efficacy and safety of a continuous subcutaneous lidocaine infusion in pediatric patients following open heart surgery.

## 2. Material and Methods

An observational prospective study was performed including all patients with an incisional lidocaine infusion in medial sternotomy after heart surgery admitted to a single Paediatric Intensive Care Unit (PICU) for two consecutive years. A total of 106 patients were included and classified according to the Risk Assessment for Congenital Heart Surgery score (RACHS1) [18]. Results were compared with a historical control group of 79 patients without incisional analgesia admitted after heart surgery between the 1st of January 2011 and the 31st of December 2011.

A catheter was inserted into the surgical incision during surgery after sternotomy closure (Figure 1(a)). An elastomeric infusion pump was used for lidocaine 0.5% infusion (Figures 1(b) and 1(c)). The infusion rate was adjusted according to the weight of the patient (Figure 1(d), Table 1).

The following demographic variables were collected: age, gender, type of heart disease and surgery, PICU length of stay (LOS), extubation in operation room (OR), time of mechanical ventilation (in hours), dose and duration of incisional lidocaine, lidocaine-related complications, intravenous concomitant sedation with midazolam or propofol, and intravenous concomitant analgesia with fentanyl, metamizole, or paracetamol. Specific scales were used to determine level of sedation (COMFORT scale) [19] and analgesia (analgesia scale, Table 2) [20]. Lidocaine levels were drawn within the first 48 hours of administration.

Data were analysed using the IBM SPSS Statistics 19 program. Qualitative variables are expressed in percentages and quantitative variables as medians and interquartile range (IQR), as variables did not follow a normal distribution. Chi-square test was used to compare qualitative variables and Mann–Whitney test to compare medians between groups. A *p* value less than 0.05 was considered statistically significant. A multivariate analysis with logistic regression adjusted for age, Risk Adjustment in Congenital Heart Surgery 1 (RACHS1) scale, and extubation in the operating room. An age-stratified analysis was also performed, with the cut-off point in two years of age.

## 3. Results

### 3.1. Characteristics of Patients with Incisional Analgesia

One hundred and six children were included in the study. Median age was 63 months (IQR 35-98 months), and 21.7% were under the age of two. Ninety patients (84.1%) were extubated after surgery in the operating room. 86% of the patients that were admitted to the PICU with mechanical ventilation were extubated within the first 24 hours of admission.

Median duration of incisional infusion with lidocaine was 48 hours (IQR 48-72). Median infusion rate was 3 ml/h (IQR 2-5 ml/h). Blood lidocaine levels were determined between 12 and 48 hours after admission in 58 patients. Blood levels were above 1.5 mcg/ml in 18 patients (31%), but none of them had levels above 5 mcg/ml. None of the patients had liver dysfunction.

Six patients (5.6%) had complications related to incisional analgesia. Three patients had catheter malposition issues and pericatheter leak which lead to early removal. The other three patients (2.8%) presented neurologic complications: A 4-month-old infant presented decreased level of consciousness and a tonic-clonic seizure. An 11-month-old patient presented decreased level of consciousness. Both had high serum lidocaine levels (3.8 and 2.4 mg/dl, respectively). Head ultrasound and 12-lead electroencephalography were normal in both patients, and neurologic manifestations disappeared after incisional analgesia was discontinued. The third patient, a 17 year-old male, presented with an acute confusional syndrome, but it was considered as not related to incisional analgesia as the infusion had been stopped a few days earlier, and blood lidocaine levels were 1.1 mg/dl. No hemodynamic adverse effects were observed throughout the study.

### 3.2. Comparison with the Control Group

Table 3 shows the comparison of patient characteristics between both groups. Children in the incisional analgesia group were significantly older, had a greater surgical risk according to RACHS1 score, and were extubated more precociously than those in the control group. Therefore, a stratified analysis was performed.

There were no differences in terms of analgesia between both groups (slight pain). Level of sedation was superficial in both groups but slightly higher according to the COMFORT scale in the incisional analgesia group (Table 3).

Fewer patients required fentanyl, propofol, and midazolam in the incisional analgesia group, and of those who did required them, doses were lower, and duration was shorter than in the control group. PICU length of stay was longer in the incisional analgesia group. Logistic regression model adjusted for age, RACHS1 score, and extubation after surgery (Table 4) confirmed the lower requirements of intravenous fentanyl in the incisional analgesia group. There were no differences in sedative drug requirements (midazolam and propofol).

### 3.3. Differences between Age Groups

Patients were divided into two groups according to age: older and younger than two years (Table 5).

In the incisional analgesia group, both age groups showed a shorter duration of intravenous fentanyl infusion than the control group. Patients older than two years required less time of fentanyl and propofol infusion as well as a lower dose of midazolam.

Median blood lidocaine levels were higher in children under two years of age (2.2 mcg/ml IQR 0.9-2.5), than in the older children (1.2 mcg/ml, IQR 0.9-1.5), *p* = 0.007. The stratified risk analysis showed that, in the incisional analgesia group, children under two had a 4.1 times greater risk of needing intravenous fentanyl than the older ones (OR 4.1; IC 95%: 1.31-12.82; *p* = 0.015). In the control group, however, there were no differences in fentanyl requirements between age groups (*p* = 0.113). The analysis did not show any differences in midazolam and propofol requirements.

## 4. Discussion

These results show that good analgesic control can be achieved with incisional analgesia after heart surgery in children, as it decreases the need for intravenous analgesic drugs. These results are consistent with previous studies in which patients with local analgesia showed better scores in pain evaluation scales than the control group in adults [14, 16] and in children [15].

A high percentage of the patients in our study required concomitant treatment with intravenous analgesic and sedative drugs, but those in the incisional analgesia group required less drugs, in lower doses and for a shorter time than those in the control group. This has also been reported in other studies [15].

Incisional analgesia is useful to control pain without increasing sedation. Level of sedation in our study, according to the COMFORT scale, was superficial in both groups but slightly higher in the control group.

The analysis of the effect of incisional analgesia in different age groups showed that the younger children needed higher doses of intravenous fentanyl. This could be interpreted as incisional analgesia being less effective in this age group. It does not seem like the doses of incisional lidocaine were insufficient because younger patients had higher blood levels of lidocaine than older children.

Assessment of pain is more complicated in infants and toddlers as it is difficult to determine whether they are crying due to pain or due to discomfort, anxiety due to separation from the parents, physical restraint, thirst, hunger, etc. Therefore, smaller children often need a combination of analgesic and sedative drugs to ensure optimal comfort. On the other hand, older children can verbally express their symptoms, so it is easier to customize treatment according to their specific needs.

The goal of incisional analgesia is to achieve local analgesia without systemic absorption, but more than 30% of our patients had blood lidocaine levels over 1.5 mcg/ml. Nevertheless, our study showed a very low incidence of adverse effects related to incisional analgesia. When lidocaine is used as an antiarrhythmic drug, goal blood therapeutic levels range between 1.5 and 5 mcg/ml. Adverse effects have been reported in literature with therapeutic lidocaine blood levels, especially in patients under three years of age [21–23]. The two patients that presented neurological symptoms were infants and had the highest blood lidocaine levels in our series (over 2 mcg/ml).

For this reason, we consider it important to monitor neurological status closely and to determine blood lidocaine levels within the first 24 hours of treatment to promptly detect patients at risk of high systemic absorption and, therefore, avoid toxicity. If neurologic manifestations appear and no other explanation is found, lidocaine toxicity must be suspected, and infusion must be stopped even if blood levels were not in the toxic range, especially in the younger patients [21].

Our study has several limitations. It is a single center study with a specific protocol for sedation and analgesia. Moreover, the control group was collected retrospectively from a historic cohort of patients, and groups were not comparable in terms of age, PICU LOS, RACHS1 score, and early extubation (in the OR). For this reason, a multivariable analysis with logistic regression adjusted for these variables was made to eliminate potential biases. Thus, randomized, multicenter clinical trials with a larger sample size are needed to confirm our results, especially in younger patients.

Our study suggests that incisional analgesia can be an effective therapeutic option in pain treatment after thoracotomy, especially in children older than two.

## 5. Conclusions

Incisional lidocaine infusion seems to be an effective therapeutic option for the treatment of pain after heart surgery in children. It reduced the need for analgesic drugs, as well as the dose and duration of intravenous opioids such as fentanyl. Despite of a low incidence of adverse effects, adequate monitoring of neurologic status and lidocaine blood levels is important in all patients. If lidocaine levels are above 2 mcg/ml or if any neurological manifestations appear, lidocaine infusion must be stopped immediately.

## Figures and Tables

**Figure 1:** Incisional analgesia: (a) incisional catheter placement after heart surgery; (b) preparation of elastomeric infusion; (c) rate of infusion; (d) required material.

**Table 1:** Rate of subcutaneous lidocaine infusion according to weight.

Weight (kg)	Rate of incisional infusion (ml/h)	Dose interval (mg/kg/h)
<20	2	0.5-2
20-50	5	0.5-1.2
>50	7	<0.7

**Table 2:** Multidimensional Assessment of Pain Scale (MAPS-revised).

Categories	0	1	2	Score
Vital signs HR and/or BP	Within baseline	More than 10% increase	More than 20% increase	
Breathing pattern	No change	Development or increase of respiratory distress	Increased respiratory distress with silent or weak cry	
Facial expressions	Relaxed	Grimace	Grimace associated with silent or weak cry	
Body movements	No movements or purposeful movements	Restless	Rigid and/or limited body movements	
State of arousal	Calm or asleep	Hyperreactive	Shut down	
Total score				

HR: heart rate; BP: blood pressure.

**Table 3:** Baseline characteristics and univariate analysis.

	Global (*n* = 185)	Control group (*n* = 79)	Incisional analgesia group (*n* = 106)	*p*
Age (months)	48 (13-83.50)	24 (8-60)	63 (35-98.25)	0.001
Gender: male (*n*, %)	107 (57.8%)	48 (60.8%)	59 (55.7%)	0.548
RACHS1 score	2 (1-4)	2 (2-3)	3 (2-3)	*0.033*
Extubation in the OR (*n*, %)	131 (70.8%)	42 (53.2%)	89 (84%)	*0.001*
Intravenous fentanyl *n* (%)	130 (70.3%)	71 (89.9%)	59 (57.3%)	0.001
Days of intravenous fentanyl	2 (1-3)	2 (1-3)	1.5 (1-2)	*0.001*
Fentanyl dose (mcg/kg/h)	1 (0.5-2)	1 (1-2)	1 (0.5-1.5)	*0.001*
Intravenous midazolam *n* (%)	51 (27.6%)	32 (40.5%)	19 (17.9%)	0.001
Midazolam dose (mcg/kg/min)	2 (1-2)	2 (1-2)	1.5 (1-2)	0.001
Intravenous propofol *n* (%)	30 (16.2%)	18 (22.8%)	12 (11.3%)	*0.044*
Propofol dose (mg/kg/h)	1.5 (1-2)	1.5 (1-2)	1.5 (1-2)	0.065
Days of intravenous metamizol	3 (2-5)	3 (2-4)	4 (2-6)	*0.001*
COMFORT scale	20.1 (18.7-22.3)	19.2 (18-21.5)	21.8 (20-23.5)	*0.001*
ANALGESIA scale	1.7 (1-2.6)	1.5 (0.97-2.77)	2 (1-2.5)	0.805
Mechanical ventilation (hours)	15.50 (6-24)	12 (6-24)	24 (3-36)	0.198
PICU LOS (days)	4 (3-6)	4 (3-4)	5 (3-8)	*0.002*

Cualitative variables are expressed in numbers and rates. Cuantitative variables are expressed in medians and interquartile ranges. Significant differences in italic characters. *n*: number of patients.

**Table 4:** Multivariate analysis with logistic regression adjusted for age, RACHS1 scale, and extubation immediately after surgery. Risk of control group over the incisional analgesia group.

Factors	Odds ratio (95% confidence interval)	*p*
Need for intravenous fentanyl	6.29 (2.48-15.97)	0.001
Intravenous fentanyl for more than 48 hours	4.30 (2.09-8.84)	0.001
Need for intravenous midazolam	1.15 (0.47-2.82)	0.762
Intravenous midazolam for more than 48 hours	0.94 (0.37-2.38)	0.900

**Table 5:** Comparison between age groups.

	Patients < 2 years		*p*	Patients > 2 years		*p*
	Control group (*n* = 42)	IA group (*n* = 23)		Control group (*n* = 37)	IA group (*n* = 83)	
Basal characteristics						
Age (months)	8.50 (5-17)	6 (4-9)	0.081	60 (48-96)	76 (53-120)	0.159
Males, *n* (%)	26 (61.9%)	13 (56.5%)	0.678	22 (59.5%)	46 (55.4%)	0.683
RACHS1 score	2 (2-2)	2 (2-3)	0,750	2 (1-3)	3 (2-3)	0.052
Extubation in OR, *n* (%)	22 (54.4%)	16 (69.6%)	0.184	20 (54.1%)	73 (88%)	0.001
Postoperative period						
COMFORT scale	19 (17.7-21.6)	22 (19.5-23.7)	0.058	19.3 (18.2-20.3)	21.8 (20-23.5)	0.001
ANALGESIA scale	1.5 (0.8-2.7)	1.7 (1.2-2.2)	0.983	1.75 (1-2.9)	2 (1-2.7)	0.971
Days of iv fentanyl	2 (1-3)	1 (1-2)	0.021	2 (1-3)	0 (0-1,5)	0.001
Fentanyl dose (mcg/kg/h)	1,5 (1-2)	1.5 (0.87-2)	0.398	1 (0.9-2)	0.5 (0.5-1.25)	0.254
Days of iv midazolam	1 (0-2)	0 (0-0,5)	0.304	0 (0-0.12)	0 (0-0)	0.792
Midazolam dose (mcg/kg/min)	2 (1-2)	2 (1-2)	0.319	3 (3-5)	5 (3-8)	0.040
Days of iv propofol	0 (0-2)	0 (0-1)	0.291	0 (0-0)	0 (0-0)	0.014
Propofol dose (mg/kg/h)	1.25 (1-2)	1.75 (1-2)	0.592	2.25 (1.25-2.87)	1 (0.75-2)	0.147
MV duration (hours)	19 (7.5-24)	19 (6-48)	0.598	8 (4-17)	24 (2-30)	0.073
PICU LOS (days)	4 (3-4)	5 (3-6)	0.039	2 (2-2)	1 (1-2.5)	0.040

IA: incisional analgesia; Iv: intravenous; OR: operating room; RACHS1 score: Risk Adjustment for Congenital Heart Surgery; MV: mechanical ventilation; PICU LOS: Pediatric Intensive Care Unit Length of Stay.

## Data Availability

All data are available upon request to the corresponding author.
